The article "Rehabilitation Brace Based on the Internet of Things 3D Printing Technology in the Treatment and Repair of Joint Trauma" was retracted in 2023. Reasons: unreliable results or conclusions; concerns about the data; concerns about the peer review.

# Rehabilitation Brace Based on the Internet of Things 3D Printing Technology in the Treatment and Repair of Joint Trauma

**DOI:** 10.1155/2021/6663892

**Published:** 2021-02-25

**Authors:** Dahua Zhang, Xiang Zhang

**Affiliations:** Department of Orthopedics, The First Affiliated Hospital of Xi'an Medical University, Xi'an, Shanxi 710000, China

## Abstract

More and more people pay attention to the printing speed and quality of 3D printing tools. In order to understand whether the 3D printing rehabilitation brace can play a role in the treatment and repair of joint trauma, we used 3D printing technology to print the rehabilitation brace and compared with the traditional rehabilitation brace. The printed parts were analyzed in detail. The experimental results prove that the rehabilitation braces made by the two methods can play a role in the repair of joint trauma. However, 3D printed rehabilitation braces can better meet the needs of patients with detailed patient data in application. The braces are more suitable, and their production speed is about 35% faster than traditional methods. Through the survey of patients and doctors, it is found that the satisfaction of patients and doctors with printed braces is above 89%, while the satisfaction with traditionally made braces is only about 60%. This shows that the rehabilitation brace based on the Internet of Things 3D printing technology has a more significant role in the treatment and repair of joint trauma, and the effect is better.

## 1. Introduction

With the continuous improvement of China's medical service system, rehabilitation medicine has been widely concerned [1]. Sports rehabilitation is an important branch of rehabilitation medicine, and it is the most popular project in the social security system. In the process of continuous improvement of rehabilitation services, the rehabilitation brace industry is developing towards productization, industrialization, and personalization, and 3D printing technology based on Internet of Things has provided great help for the development of rehabilitation support [2]. 3D printing technology can be traced back to the late 1980s. It is a complete manufacturing technology with a new way of thinking and has since gradually emerged. 3D technology is a new technological form based on software technology, mechanical processing technology, special processing technology, small molecule technology, and electronic and electrical technology. [3]. 3D printing technology is a revolution of traditional manufacturing technology, which provides a new platform for its development; it is an advanced manufacturing technology used to form entity [4]. In the process of forming entity, 3D model created in advance in computer is transmitted to 3D printer through certain file format and directly produced by material stacking method.

Compared with the traditional processing and manufacturing technology in the past, 3D printing technology can not only realize “from scratch,” save a lot of time and labor, but also carry out “personalized manufacturing,” making the product unique [5]. At present, the 3D printing technology is widely concerned by the industry and has been well applied in the experimental demonstration of new product development stage, rapid mold making, direct production of small batch of special complex parts [6], application field of bioengineering, and development of new materials. In terms of design innovation, the technology can realize abstract and complex ideas quickly; it can manufacture according to the type, save materials, and reduce energy consumption; it can express the rapid manufacturing process of personalized products in the form of graphics and animation and show the trend of people's pursuit of diversified and personalized products in the future [7]; it can use the form of graphic and graphic cases to show the rapid manufacturing process of personalized products; it has the function of integrated design and optimized design and manufacturing with shape. There are also many researches on the rehabilitation brace of 3D printing technology at home and abroad [8].

Liu Zheng thinks that the traditional rehabilitation brace manufacturing process is complex, and the accuracy is difficult to adapt to the patients and meet the needs of patients. Therefore, it is very important to use 3D printing technology to make rehabilitation support. 3D printing technology can print the rehabilitation support into a structure and shape suitable for patients according to the patient's situation. Qiang combined 3D printing technology with traditional rehabilitation technology, innovatively proposed the shape and appearance design of 3D technology in rehabilitation brace, introduced the difficulties and challenges faced in the application of 3D printing technology in practice, elaborated the important role of 3D printing in promoting the integration of medical and engineering technology, and highly praised the value of 3D printing technology in rehabilitation brace [9, 10]. Zhengwen introduced the development history and prospect of rehabilitation brace at present. He believed that the medical devices made by 3D printing technology could provide convenience for people. In this paper, the printing method and principle of 3D printing technology were introduced in detail, and the characteristics and advantages of printing products were also explained. The application and problems of 3D printing technology in medical treatment in China were summarized; the future development direction is also discussed. These studies have some advantages, but there are also some deficiencies. The data of the research are too limited, and there is few experimental support, which can only provide some theoretical reference.

In this paper, through the establishment of 3D printing rehabilitation brace model, it is compared with the traditional rehabilitation brace in all aspects, to test whether it can play a role in joint trauma. Collect relevant experimental data to analyze the comparison results of the experimental data in detail. Finally, patient and expert reviews can conclude that the results supporting 3D printing repairs have high practical value.

## 2. Internet of Things 3D Printing Rehabilitation Support Printing

### 2.1. Internet of Things

The Internet of Things is a complex system in many forms and includes many areas of social life [11]. Although the structure of the IoT system is complex and the functions and scales of different IoT application systems are very different, they must have many inherent common characteristics. With reference to how to explore mature computer network architecture models, the Internet of Things is divided into recognition, network, and application levels. The Internet of Things is a combination of the Internet and various information retrieval devices that connect people to everything and everything to everything [12]. The design principles of the Internet of Things supply chain management system should cover the following aspects [13].

1. *The Principle of Appropriateness*. The principle of appropriateness refers to the fit between the supply chain management system based on the Internet of Things and the characteristics of the supply chain itself. As a new generation of information technology, the Internet of Things technology is regarded as the third wave of information technology and the key to grasp the competitive advantage of the information industry in the future. However, for the decision-makers in the supply chain, the realization of interests is the main goal, and the advanced technology should be treated calmly and objectively instead of blindly worshipping; only the supply chain management system which is consistent with the characteristics of the supply chain itself is the most reasonable and appropriate system. Any reasonable system must conform to the principle of cost and benefit. The construction of supply chain management system based on the Internet of Things technology must also conform to the principle of cost and benefit [14]. Particularly for the decision-makers in the supply chain, they should be based on their own resources and funds, not on the interests of the core enterprises.
2. *Expansibility Principle*. The principle of scalability refers to the difficulty of developing new functions of supply chain management system based on the Internet of Things technology and connecting with new technologies in the future under the environment of Internet of Things. As the third wave of information technology, the Internet of Things has the characteristics of real time and interaction. Therefore, the development of the Internet of Things is bound to be in constant change. Therefore, the supply chain management system based on the Internet of Things should also be adjusted in real time according to the continuous development of the Internet of Things technology [15]. A kind of management system needs to pay huge manpower, material resources, financial resources, time, and other resources from the concept generation to the formation and application, and different management systems have the characteristics of path dependence, which also leads to its high conversion cost. Therefore, when constructing the supply chain management system based on the Internet of Things, it is necessary to have the foresight thinking, judge the development trend of the future Internet of Things technology in advance, and reserve relevant interfaces for docking, so as to avoid or minimize the adjustment of the supply chain management system when the future technology continues to develop [16].
3. *Reuse Principle*. The principle of reuse means that the supply chain management system based on the Internet of Things should have certain universal applicability, and it should have a standard core in terms of function and structure, which can be applied to different supply chains with slight or no adjustment. As the carrier of the Internet of Things technology, the supply chain can play the same role at different scales, i.e., to improve the transparency and visibility of the entire supply chain, to improve the stability of the entire supply chain, and to improve its intelligence level supply chain. Therefore, similar carriers can be replicated between supply chains with little or no adjustment. According to the different carriers, adjust and expand the application according to their scale and function. Therefore, the principle of reuse has been implied in the design principles of supply chain management system based on the Internet of Things [17].
4. *The Principle of Voluntary Coordination and Cocreation*. The supply chain based on the Internet of Things includes multiple decision-makers and stakeholders. The management of the supply chain needs to be completed through mutual consultation and cooperation. The main goal of the supply chain management system based on the Internet of Things is to reduce the uncertainty of the supply chain, improve the visualization level of the supply chain, increase the transparency of the supply chain, and improve the intelligence level of the supply chain. To achieve this goal, we need to invest a huge cost, which requires the joint efforts of all decision-makers in the supply chain. As downstream enterprises need to implement the Internet of Things strategy based on the upstream enterprises, there is a free ride for downstream enterprises, which will inevitably lead to the uneven cost input and benefit distribution of each decision-making body in the supply chain, damage the interests of relevant decision-makers in the supply chain, and affect their enthusiasm [2]. In addition, the core enterprises in the supply chain play a key role in the whole chain, and their strategy adjustment in the supply chain will directly or indirectly force the enterprises in the supply chain to adjust, which makes the smooth progress of the whole supply chain have potential risks. Therefore, the supply chain management system based on the Internet of Things should design a relevant interest coordination mechanism to share various costs and interests and improve the enthusiasm of decision-makers [18].

### 2.2. 3D Printing Technology

Generally speaking, it is an important problem in the field of 3D printing to improve the printing accuracy and printing efficiency at the same time. If you want to improve the printing efficiency, the printing accuracy will certainly decline. No matter which method is used to make the model directly 3D printing, dimensional accuracy and surface roughness are key parameters [19]. The 3D printing process is as follows: 3D CAD modeling ⟶ computer layered processing of CAD model ⟶ layer information processing ⟶ layer manufacturing and connection ⟶ finally printing the part model. All processes have a direct impact on the accuracy of the model. The mold is generally expressed by the following formula when printing:

(1) $$\begin{array}{c} r=\frac{\text{pnd}}{\lambda },\\ N=0.25r^{0.8}{\mathrm{Pr}}^{0.4},\\ \frac{\alpha *d}{\sigma }=0.25{\left(\frac{d*r*p}{\kappa }\right)}^{0.8}{\left(\frac{c*u}{\sigma }\right)}^{0.4}. \end{array}$$

After the above formula is simplified,

(2) $$\begin{array}{c} \alpha =\frac{2.057f*{\left(v*p\right)}^{0.8}}{d^{0.2}}. \end{array}$$

Since the emergence of 3D printing technology, there are more than ten kinds of processes. At present, there are several typical commercialization processes.

#### 2.2.1. UV Curing Molding Technology

Stereolithography technology, also known as stereolithography technology, is a rapid prototyping manufacturing process with the earliest development, the most mature technology and the most widely used in the world. Based on the principle of light curing of liquid resin materials, UV light or laser is used as the light source to gather the laser beam into a spot with a diameter of about 0.1 mm. Depending on the movement of the reflected galvanometer, the laser beam is guided to focus on the surface of the UV curable material, which is solidified layer by layer in the order of point, line, and surface. After curing one layer, the worktable rises one layer of thickness along the *z-*axis, and then another layer is solidified. Finally, the model entity is obtained by stacking layer by layer [20]. The advantages of UV curing molding process are high precision, which can reach 0.016 mm; good surface quality; the utilization rate of raw materials is close to 100%; and it can print out small parts with complex shape. The disadvantage is that the cost of UV curing molding equipment and printing consumables is high; the molding entity is mainly resin materials, with poor stiffness, strength, oxidation resistance, and heat resistance, which is not easy to be preserved for a long time.

#### 2.2.2. Lamination Molding Technology

Laminated molding technology is to use coated paper, coated ceramic film, metal foil, plastic foil, and other materials; one side of these materials is precoated with a layer of hot melt adhesive. In the printing process, the materials are heated by the heating roller and bonded together. The two-dimensional profile data obtained from the laser beam cutting model is used to cut the material. Then, the new material layers are stacked together, and then the new material layers are glued together. This process is repeated until the entire part is formed [21]. Laminated molding technology is suitable for conceptual modeling of product design and functional testing of parts, especially for direct manufacturing of sand mold. Lamination technology has the advantages of high hardness, good mechanical properties, short molding time, high molding efficiency, and low cost. The disadvantage is that the precision of forming surface is not high, and the tensile strength and elasticity of printed parts are not good.

#### 2.2.3. Melt Deposition Molding Technology

The melt deposition forming technology is to send the filiform material to the nozzle and heat it to the semi-flow state. The CAD model is divided into several layers of slices by the layered software. The molten material solidifies rapidly, layers are piled up and bonded tightly, and the part model is finally obtained. In FDM machines, the middle height is determined by the diameter of the extruded wire, usually from 0.15 mm to 0.25 mm, which represents the best tolerance range that can be achieved in the vertical direction [22]. In the *XY*-plane, the control accuracy of the motor can reach 0.025 mm, but due to the diameter of the extruded wire, the machining accuracy of FDM equipment is generally only 0.3 mm. FDM has the advantages of clean printing process, strong operability, and low garbage generation. The disadvantages are that the precision of the printed products is low, the surface has obvious layered stripes, the support structure needs to be formed at the same time, and it is not suitable for printing parts with excessively complex structure. The materials used in FDM process are usually thermoplastic materials, such as ABS, PLA, wax, artificial rubber, etc.

#### 2.2.4. Selective Laser Sintering Technology

Selective laser sintering (SLS) technology uses high-intensity laser emitted from CO2 laser to sinter powder materials such as plastics, paraffin, metal, and ceramics in layers and solidify them layer by layer and then form three-dimensional objects after stacking. During the work, the powder material is evenly spread on the upper surface of the formed parts by the powder laying system, and the computer transforms the two-dimensional profile data information after slicing into the irradiation track of high-intensity laser beam. The material powders are selectively sintered together to form a layer of cross section of the printing part and connected with the solidified part below. After a layer of powder is sintered, a layer of powder is laid in the powder laying system and then sintered. The process is repeated and accumulated layer by layer, and the part model is obtained. The advantages of SLS process are that the strength and mechanical properties of parts are higher after forming; there is no need for design and construction support; there are many kinds of materials available [23]; and the utilization rate of raw materials is close to 100%. The disadvantage is that it needs a special workshop filled with flame retardant gas such as nitrogen, which has high cost of use and maintenance; the material needs to be heated and preheated before processing and needs to be cooled for a long time after molding, so the molding efficiency is low; the surface of the molded parts is loose and porous, so it needs to carry out complex posttreatment; there is odor in the sintering process, which pollutes the environment. The 3D printing process is shown in Figure 1.

### 2.3. Rehabilitation Support

With the continuous improvement of science and technology research and development ability, the substitution rate of domestic low-end rehabilitation brace for imported products has exceeded 90%. Due to the backwardness of core technology, high-end scientific research and comprehensive equipment still rely on imports. Rehabilitation support industry is looking for the transformation from special equipment and tools to industrial production. Compared with the design pain points of traditional medical devices, such as functional output, complex operation, and debugging, rehabilitation brace has been able to achieve private customization and formed an industrial scale. Therefore, user experience plays an important role in the design of knee rehabilitation brace.

The design and development process of rehabilitation brace products should pay special attention to the safety design of safety, function, structure, shape, human-computer interaction, and psychology. The nonstandardized design process of medical devices will lead to many unknown errors of operators and users: the medical accidents caused by the lack of adequate training account for 70% to 90%. Poor medical devices make it more difficult for professionals to train, and many patients lose their confidence in medical devices because of the trouble in operation and lack of care for patients, so they choose expensive artificial rehabilitation services instead. Therefore, both doctors and patients are eager to have well-designed rehabilitation support products, which can effectively reduce the probability of accidents in operation. The safety design of assistive devices is not only the design of “things,” but also the design of “people” [24].

The design features of medical devices and traditional rehabilitation braces are similar. Both of them belong to activity-centered interactive design or system design. They are mainly developed for technical realization and function realization. In today's medical environment and actual rehabilitation treatment, how to fully understand and transform users' expectations and needs, how to fit the shape, structure, and function of the product to the needs of users is the key point in the design process of rehabilitation support; that is, the design of rehabilitation support urgently needs the guidance of user research design decision [25]. When the ratio of the length to the wall thickness of the brace is greater than 10, the brace is regarded as a thin-walled part

(3) $$\begin{array}{c} \frac{\partial z}{\partial t}=\alpha \frac{\partial^{2}z}{\partial n^{2}},\\ Q=\frac{\gamma }{t}A_{n}\left(T_{m}-T_{n}\right),\\ q=\beta *\partial *\left[{\left(\frac{t_{1}}{100}\right)}^{4}-{\left(\frac{t_{2}}{100}\right)}^{4}\right]. \end{array}$$

The product users of joint rehabilitation brace are divided into two user groups: (1) direct users: the patient group, the direct users need to contact with knee joint rehabilitation aids directly and directly experience the functions provided by rehabilitation aids. In case of discomfort, abnormal equipment, and other situations, doctors and family members need to be informed in time to ensure the normal use of the equipment and prevent the equipment from causing secondary injury to the affected area. (2) Expert users: doctors, before the use of the device to guide patients and inform the precautions, adjust the equipment according to the patient's body size, and set the parameters of the equipment according to the patient's pathology and use history. It is necessary to monitor the use status of patients within a certain range, collect the feedback information of patients, and timely adjust the equipment or deal with emergencies [26].

Joint rehabilitation brace is a special equipment product rather than a common consumer product. The research identified the product trend of rehabilitation brace, focused on the design of knee joint rehabilitation assistive device, conducted product research and analysis based on rehabilitation course, found the design opportunity point of knee joint rehabilitation brace, and defined the design direction [27]. A comprehensive understanding of the expectations and needs of the target user group is the key to the success of product design. The users of knee joint rehabilitation brace are divided into two user groups: patients and rehabilitation doctors. As designers, it is difficult to carry out demand reasoning based on their own knowledge and experience. After analyzing and classifying the users of the product, we focus on obtaining the user requirements in the user research process, which plays a guiding role in the selection and decision-making in the product design process [28].

### 2.4. Application of Rehabilitation Brace Model

The support model is parameterized and then transmitted to the data model. The data module receives the needs of users, finds appropriate resources through resource evaluation, performs tasks, and completes user requests [29].

Considering the resources with the same service function, the attributes of the resources are set according to the user preferences and have certain scalability [30]. The calculation formula is as follows:

(4) $$\begin{array}{c} U_{a}=p*b\frac{j}{i}*c. \end{array}$$

In order to calculate the attribute weight and ensure the objectivity of the evaluation results, we use the entropy weight method to determine the entropy value and entropy weight of each resource attribute.

(5) $$\begin{array}{c} t=\frac{1}{\ln\;x}\sum_{n=1}^{1}f_{nm}*\;\ln\;f_{nm},\\ r=\frac{1-t}{y-\sum_{m=1}^{m}t},\\ f_{mn}=\frac{z_{nm}}{\sum_{n=1}^{x}z_{nm}},\\ \sum_{m=1}^{x}w_{m}=1. \end{array}$$

Set objective weights for each user attribute:

(6) $$\begin{array}{c} d=\sqrt{\sum_{m=1}^{x}w_{n}*{\left(r_{nm}-uq_{m}\right)}^{2}},\\ d_{n}=\frac{1}{1+d\left(r_{n},uq\right)}. \end{array}$$

Set the proximity threshold value between [0,1], from which the matching value *Q* can be obtained:

(7) $$\begin{array}{c} Q_{\delta }=\left\{r_{n}\left|d\;\cos\left(r_{n},uq\right)\right|\geq \delta \right\}. \end{array}$$

The simulation parameters are calculated as follows:

(8) $$\begin{array}{c} F=\frac{\sum \left(q_{rp,rpn}-q_{rpm}\right)\left(q_{uq,uqn}-q_{uq}\right)}{\sum_{n=1}^{n}{\left(q_{r}-q_{uq}\right)}^{2}\sqrt{\sum {\left(q_{uq,uqm}-q_{uq}\right)}^{2}}}. \end{array}$$

## 3. Application of Rehabilitation Brace in the Treatment of Joint Trauma

### 3.1. Purpose of the Experiment

In this paper, based on the theoretical results of the Internet of Things 3D printing research, using the methods of literature, comparative research, mathematical statistics, logical analysis, and other methods, this paper analyzes the application of rehabilitation brace and the difference between 3D printing and conventional production and studies its application mode and characteristics.

### 3.2. Experimental Evaluation Criteria

We investigated 100 doctors and 100 patients and asked them to score the rehabilitation brace. The score was divided into four stages, and the score was carried out according to the entropy method.

Entropy method is a relatively objective evaluation index weight assignment method, which can effectively avoid the subjectivity of artificial scoring, and has high accuracy. But at the same time, this study also realized that the entropy method cannot directly reflect the knowledge, opinions, and experience judgment of experts and scholars, and the weight results may be contrary to the actual situation. Therefore, this paper uses AHP and entropy method to determine the weight coefficient of regional higher education evaluation index.

*Comprehensive Quantitative and Qualitative Analysis*. Quantitative analysis is to analyze the data of the problem, using the intuitive and clear essence of mathematics to reflect the existence of the problem; qualitative analysis is to collect, read and sort out the relevant domestic and foreign research literature, and systematically summarize the relevant theoretical results. Some standards cannot be directly analyzed by quantitative method but can only be evaluated by qualitative analysis. The evaluation standard system is constructed by combining quantitative and qualitative analysis methods. At the same time, the calculation formula and evaluation standard of relevant standards are given.

### 3.3. Data Sources

In this paper, Internet of Things, 3D printing, rehabilitation brace, etc., are used as keywords, and the starting and ending years are set as 2015–2019. The relevant literature is searched by CNKI, Baidu, and other network platforms, and the collected data are classified and sorted. 167 Chinese and foreign academic papers, 29 academic works, 34 newspapers and network materials, and 15 doctoral and master's theses related to this research are obtained. At the same time, through questionnaire survey and field interview, we collected the opinions of patients and doctors on 3D printing rehabilitation brace and traditional rehabilitation support.

## 4. Experimental Analysis of Rehabilitation Brace in Joint Trauma Repair

### 4.1. Comparison of Rehabilitation Brace Effect

We have made statistics on the use effect of 3D printing rehabilitation brace (control group) and traditional rehabilitation support (experimental group) by doctors and patients. The specific data statistics are shown in Table 1.

It can be seen from Figures 2 and 3 that both doctors and patients recognize the role of rehabilitation brace in joint repair. More than 70% of the people think that rehabilitation brace can play a role in joint trauma repair, and about 30% of them give more than 90 points and think that it can play a very important role. In particular, the rehabilitation brace using 3D printing technology is more important in the eyes of patients and doctors, and more braces with 3D printing score above 75 account for more.

### 4.2. Comfort of Rehabilitation Brace

We investigated the feelings of patients and doctors after using rehabilitation brace and counted their opinions on the use of 3D printing rehabilitation brace and traditional rehabilitation brace. The specific statistical data are shown in Table 2.

From Figures 4 and 5, we can see that, in this survey, doctors and patients have similar views on the comfort degree of the brace. The overall comfort level of the traditional brace survey is about 50%, while that of the 3D rehabilitation brace is more than 70%. This is because the 3D printed rehabilitation brace is made according to the personal data of the patient. If the support is suitable, the evaluation will be higher.

### 4.3. Support Fabrication Speed

We have made statistics on the time required for 3D printing rehabilitation brace and traditional rehabilitation brace. Relatively speaking, in a small amount of cases, the time required for 3D printing and traditional rehabilitation brace is similar. However, in mass production, the production speed of 3D printing is extremely excellent. The specific data are shown in Table 3.

From Figures 6 and 7, we can see that the overall speed of 3D printing is better than that of traditional manufacturing methods. In single and batch production of 3D printing rehabilitation brace, the speed changes little, from 197 minutes to 253 minutes on average. However, there is little difference between the time consumed by traditional methods and printing when a small amount of rehabilitation braces are made by traditional methods, but when multiple batches are made, the time required is greatly different, which is due to the difference between manual and mechanical.

### 4.4. Success Rate of Production at the Time of Rehabilitation

The production of rehabilitation brace requires a lot of materials and time, so it is very necessary to maintain a high success rate of brace fabrication. However, there is a certain risk of failure in both 3D printing and traditional production. Overall, the success rate of 3D printing is higher than that of traditional production. The specific data are shown in Table 4.

As can be seen from Figure 8, the overall printing success rate of rehabilitation brace is about 90%. With the increase of the length of support, the success rate of traditional printing method gradually decreases, which is due to the fatigue of human resources under long-term work. However, the success rate of 3D printing has little change, and the overall success rate is nearly 10% higher than that of traditional production, which shows that 3D printing production is better than traditional production in the production of rehabilitation support.

## 5. Conclusions

3D printing based on virtual reality is based on the 3D CAD model created by 3D design software. The 3D digital model is divided into two-dimensional slicing models with several layers by the software. The contour information of these two-dimensional slice models is imported into the 3D printer to convert it into the moving track of the printing head. The special materials such as liquid, cell tissue, plastic, powder, etc., can be transformed into the moving track of the printing head. Finally, a solid body is formed by layer superposition and bonding by melt nozzle and laser beam.

Through prototype design, production and debugging, and product modeling design, the design decision is implemented on the product. The process of joint rehabilitation brace product development was completed from investigation analysis, user research, demand acquisition, design decision, design, and development. Through the analysis of the special user group of rehabilitation support equipment, the reasonable user research method is selected, and the user research route in the design and development process of rehabilitation support equipment is summarized.

In this paper, user interviews and user behavior observation methods are used to obtain user requirements. These methods are subjective. In the follow-up research process, we will use physiological signal measurement equipment, behavior analysis model analysis tools, product user test, and other quantitative attribute tools and research methods to conduct design research, information acquisition, and product verification, so as to improve the quality of user research.

## Figures and Tables

**Figure 1:** 3D printing process.

**Figure 2:** Patient data statistics.

**Figure 3:** Doctor data statistics.

**Figure 4:** Comfort survey of brace.

**Figure 5:** Comfort of different supports.

**Figure 6:** Support fabrication speed.

**Figure 7:** Time required for support fabrication.

**Figure 8:** Time required for support fabrication.

**Table 1:** Effect of rehabilitation brace.

		0–60	60–75	75–90	90–100
Patient	Experience group	13	34	37	16
	Control group	2	17	41	40

Doctor	Experience group	17	21	47	15
	Control group	6	9	59	26

**Table 2:** Comfort of rehabilitation brace.

		Discomfort	Commonly	Comfortable	Very comfortable
Patient	Experience group	10	41	34	15
	Control group	2	24	35	39

Doctor	Experience group	8	34	37	21
	Control group	3	19	42	36

**Table 3:** Production time of rehabilitation brace.

	1 (min)	5 (min)	10 (min)	15 (min)	20 (min)
Traditional hand brace	221	235	235	259	272
Traditional leg brace	198	217	231	247	269
Traditional prognostic brace	341	357	369	378	385
3D printing hand support	178	189	196	207	211
3D printing leg brace	186	199	204	217	226
3D printing prognosis support	265	278	286	299	317

**Table 4:** Production time of rehabilitation brace.

	50 cm (%)	100 cm (%)	150 cm (%)	200 cm (%)
Traditional hand brace	89	87.50	82.70	81.90
Traditional leg brace	91.50	90.70	92.40	89.70
Traditional prognostic brace	90.70	89.60	88.40	86.70
3D printing hand support	95.40	94.90	93.70	92.60
3D printing leg brace	93.70	93.20	92.70	92.40

## Data Availability

No data were used to support this study.
